The article "Comparative Study on the Clinical Efficacy and Safety of Acitretin and MTX in the Treatment of Pustular Psoriasis by TLR7/MyD88/CXCL16 Pathway" was retracted in 2023. Reasons: signs of a paper mill; suspected computer-generated content; unreliable results or conclusions; concerns about the data.

# Comparative Study on the Clinical Efficacy and Safety of Acitretin and MTX in the Treatment of Pustular Psoriasis by TLR7/MyD88/CXCL16 Pathway

**DOI:** 10.1155/2022/9640326

**Published:** 2022-03-18

**Authors:** Jiajing Lu, Yu Wang, Ying Li, Yu Gong, Yangfeng Ding, Yuling Shi

**Affiliations:** ^1^Department of Dermatology, Shanghai Skin Disease Hospital, School of Medicine, Tongji University, Shanghai 200443, China; ^2^Institute of Psoriasis, School of Medicine, Tongji University, Shanghai 200443, China

## Abstract

**Objective:**

To investigate the clinical efficacy and safety of acitretin and MTX with TLR7/MyD88/CXCL16 in the treatment of pustular psoriasis.

**Method:**

A total of 54 patients with pustular psoriasis were randomly divided into control group (*n* = 14) and study group (*n* = 40). MTX was used in the control group, and different doses of acitretin were used in the study group, which were divided into low-dose group (*n* = 13), medium-dose group (*n* = 13), and high-dose group (*n* = 14). Symptom relief time, recurrence rate, GPPASI improvement rate, treatment response rate, BSA, DLQI score, and TLR7 and CXCL16 levels were compared among four groups.

**Result:**

The erythema, fever, and pustules disappeared in the low-dose group, the medium-dose group, and the high-dose group for a shorter time than control group, and it is shortest for the high-dose group. The low-dose, medium-dose, and high-dose groups had relatively lower recurrence rates at 1 month and 3 months (*P* < 0.05). The improvement rates of GPPASI50 of the four groups (the control group, low-dose group, medium-dose group, and high-dose group in turn) were 71.4%, 78.3%, 80.2%, and 80.8%; GPPASI75 of the four groups were 73.5%, 74.3%, 79.4%, and 80.9%; and GPPASI90 were 12.9%, 13.1%, 13.4%, and 13.8%. After treatment, the BSA and DLQI scores of the four groups were reduced. The BSA and DLQI scores of the study group decreased more significantly, and the high-dose group had the most significant improvement (*P* < 0.05). The incidence of adverse reactions in the four groups was 16.2%, 8.1%, 10.3%, and 14.7%, respectively. The high-dose group had a higher incidence of adverse reaction than the low-dose group (*P* < 0.05). The effective rates of treatment of the four groups were 69.1%, 86.9%, 88.2%, and 91.9%, respectively. The study group had higher treatment efficiency than the control group, and the high-dose group had the highest treatment efficiency (*P* < 0.05). After treatment, the level of serum TLR7 and CXCL16 was significantly reduced, but which in the study group decreased more significantly (*P* < 0.05).

**Conclusion:**

The clinical effect of a high dose of acitretin on pustular psoriasis is remarkable. It can reduce the recurrence rate and improve the quality of life and clinical symptoms. Therefore, a high dose of acitretin is worth popularizing and applying.

## 1. Preface

Psoriasis involves 125 million people worldwide, and there are about 6.5 million psoriasis patients in China [1], among which pustular psoriasis accounts for 0.69% of all psoriasis patients [2], and it is increasing year by year. Japanese data shows [3]the following: generalized pustular psoriasis (GPP) patients accounted for 1.2% of psoriasis patients and the incidence of GPP in the Asian population is as high as 7.46/million. The incidence and prevalence of GPP in France in 2004 was 0.64 per million and 1.76 per million, respectively, with complications in 17% and mortality in 2% [2]. Pustular psoriasis can affect the skin and multiple systems. The application of acitretin treatment can bind to the corresponding receptors to regulate cell proliferation and differentiation, can resist microvascular formation, and is a pharmacologically active metabolite of acitretin. Acitretin has the characteristics of relatively low side effects, high availability, low accumulation, and short half-life. It is very important in the treatment of pustular psoriasis, plaque psoriasis vulgaris, and erythroderma psoriasis [4]. In this study, 54 patients with pustular psoriasis admitted to our hospital were treated with different doses of acitretin and MTX to compare the treatment effect and safety of patients with pustular psoriasis, explore appropriate treatment plan, improve the efficiency of diagnosis and treatment, and improve the quality of life to a greater extent. The report follows.

## 2. General Information

A total of 54 patients with pustular psoriasis were randomly divided into control group (*n* = 14) and study group (*n* = 40). We use MTX for the control group, and different doses of acitretin was used for the study group and divided into three groups: low-dose group (*n* = 13), medium-dose group (*n* = 13), and high-dose group (*n* = 14). In the control group, there were 7 males and 7 females, from 20 to 65-year-old, with an average age of 52.8 ± 4.5. In the study group (*n* = 40), there were 21 males and 19 females, from 20- to 65-year-old, with an average age of 52.6 ± 4.4. The research subjects agreed with the study, the data were comparable (*P* > 0.05), and the hospital ethics committee agreed with the study.

Inclusion criteria are as follows [5]: (1) Patients are from 18 to 65-year-old. (2) Patients with a course of disease more than 6 months. (3) Clinically diagnosed patients with pustular psoriasis. (4) Patients with normal cognitive function, who can cooperate with the study. (5) Patients who did not receive calcineurin inhibitors, vitamin D3 derivatives, glucocorticoids, and systemic therapy, etc. 15 days before the study. (6) Patients with stable vital signs and acceptable prognostic follow-up. Exclusion criteria are as follows: (1) Patients with allergy or intolerance to the study drug. (2) Patients with a history of severe allergic reactions. (3) Patients with malignant tumors, autoimmune diseases, or systemic diseases. (4) Patients during lactation, pregnancy or planning to become pregnant. (5) Patients who received topical medication and systemic therapy 15 days before the study.

## 3. Method

1. The control group was given MTX (National Drug Approval: H20080251, manufacturer: Shanghai Xinyi Pharmaceutical Co., Ltd.) at a dose of 10 mg/week, which was maintained until the 52th week. Drug resistance was assessed during the treatment and follow-up after continuous rain was performed
2. The study group was given different doses of acitretin (national drug approval H20010126, manufacturer: Chongqing Huabang Pharmaceutical Co., Ltd.). (1) The low-dose group was 0.3 mg/kg/d, maintained to 52 weeks. (2) The medium-dose group was 0.4 mg/kg/d, maintained to 52 weeks. (3) The high-dose group: 0.5 mg/kg/d, maintained to 52 weeks. The drug resistance of patients was evaluated during treatment, and follow-up after continuous prognosis was carried out, and the treatment plan was adjusted appropriately according to the treatment situation

### 3.1. Observation Index

Time to resolve symptoms: count the time to resolve erythema, fever and pustules.

Recurrence rate: count the number of recurrence and non-recurrence cases, and calculate the incidence rate.

GPPASI improvement rate [6]: the situation of erythema (E), pustules (P), desquamination (D), and affected area(%)were evaluated by GPPASI scoring system. 0 points: no erythema, visible pustules, and desquamation. 1 point: almost no erythema, pustules and desquamation. 2 points: Slight erythema, pustules, and desquamation. 3 points: moderate erythema, pustules, and desquamation. 4 points: severe erythema, pustules, and desquamation. The affected area was from 0% to 100%. Note: GPPASI = (E + P + D) × affected area × 0.1(head) + (E + P + D) × affected area × 0.2(upper limbs) + (E + P + D) × affected area × 0.3(truncus) + (E + P + D) × affected area × 0.4(lower limbs).

BSA and DLQI score [7]: BSA score means area of body surface involvement, slight < 3%, moderate 3% ~ <10%, and severe ≥ 10%. The dermatological quality of life index (DLQI) is used to evaluate life quality patients, including treatment impact, pain or itching, sexual disturbance, feeling distressed, relationship with friends or family, daily activities, work and/or study, dress, exercise, 10 questions about social life, 0-3 points for each item.

Adverse reactions: count the number of cases of itchy skin, dry skin, desquamation, chapped lips, dry eyes, mild headache, elevated triglycerides, elevated cholesterol, gastrointestinal discomfort, leukopenia and abnormal liver function, and calculate the incidence.

Effective treatment rate: ineffective: GPPASI regression is less than 25%; effective: GPPASI regression is between 25% and 69%; markedly effective: GPPASI regression is greater than 69%. Effective rate = (markedly effective + effective) number of cases/total number of cases × 100%.

Level of TLR7 and CXCL16: 3 mL of fasting venous blood was extracted and centrifuged at 3500 RPM to obtain serum. ELISA was used for detection. Relevant operations were carried out according to the instructions.

### 3.2. Statistical Method

We enter the collected data into the EXCEL form and use the statistical SPSS22.0 software for data analysis. We carry out a normal distribution test on the collected data. If the data conform to a normal distribution, the count data shall be described by composition ratio and rate. The chi-square test will be used to analyze groups' difference, and measurement data shall be expressed as mean ± standard deviation. The *t* test was used to analyze groups' difference. The physical influencing factors of the case group were analyzed by logistic regression, and *P* < 0.05 was taken as the difference was statistically significant. The graph software used by the institute was GraphPad Prism 8.

## 4. Result

### 4.1. Time to Symptom Resolution

When comparing with the control group, the erythema, fever, and pustules disappear in the study group for a shorter time. The difference between the groups was significant in statistical analysis (*P* < 0.05) (Table 1).

### 4.2. Recurrence Rate at 1 Month and 3 Months

When comparing with the control group, the study group had lower recurrence rates at 1 month and 3 months. The difference between the groups was significant in statistical analysis (*P* < 0.05) (Table 2).

### 4.3. Improvement Rates of GPPASI50, GPPASI75, and GPPASI90

When comparing with the control group, the improvement rates in GPPASI50, GPPASI75, and GPPASI90 of the study group were greater, and from low to high were low-dose group, medium-dose group, and high-dose group, respectively. The difference between the groups was significant in statistical analysis (*P* < 0.05) (Figure 1).

### 4.4. BSA and DLQI Scores

The BSA and DLQI scores of the four groups were no significant difference before treatment and were significantly reduced after treatment, and it decreased more significantly in the study group, with the high-dose group improved the most. The difference between the groups was significant in statistical analysis (*P* < 0.05) (Figure 2).

### 4.5. Incidence of Adverse Reactions

The incidence of adverse reactions in the four groups was 16.2%, 8.1%, 10.3%, and 14.7%, respectively. When comparing with the other two study groups, the high-dose group had a higher incidence of adverse reactions, the difference was significant in statistical analysis (*P* < 0.05) (Figure 3).

## 5. Treatment Efficiency

The effective rates of treatment in the four groups were 69.1%, 86.9%, 88.2%, and 91.9%, respectively. Comparing with the four groups, the difference was significant in statistical analysis (*P* < 0.05) (Figure 4).

### 5.1. Level of TLR7 and CXCL16

After treatment, the level of serum TLR7 and CXCL16 was reduced. Comparing with the four groups, the difference was significant in statistical analysis (*P* < 0.05) (Table 3).

## 6. Discussion

Psoriasis is an inflammatory, chronic, and recurrent disease. Pustular psoriasis is a severe and refractory type, and its clinical treatment is extremely challenging. Therefore, a reasonable and standardized treatment plan should be formulated according to the specific conditions of patients [8, 9].

At present, there are more and more researches on skin immune diseases, but most patients will choose traditional medicine treatment in the medical insurance catalog, and only a few patients will choose biological treatment [10]. In this study, acitretin was selected to treat pustular psoriasis with long lasting effect. It is the second-generation retinoic acid drug. The main mechanism of the drug treatment is as follows: (1) It has a regulatory effect on the terminal differentiation of keratinocytes and inhibits abnormal proliferation. In turn, it can alleviate symptoms such as nail hypertrophy and excessive subungual keratosis [11]. (2) It can reduce the cohesion and the permeability barrier function of the stratum corneum, which can significantly improve the penetration of drugs [12]. (3) It plays the role of inhibiting inflammation and immune regulation and can regulate the activation of lymphocytes [13, 14]. In turn, it inhibits the secretion of inflammatory mediator factors, weakens the chemotaxis of neutrophils, reduces leukotrienes and oxidized anions, inhibits the production of inflammatory arachidonic acid and metabolites, reduces inflammation, and reduces nail damage [15]. (4) It will downregulate the expression of ROR*γ*tmRNA in peripheral blood, increase the expression of Foxp3mRNA, reduce the release of IL-17 factor, and achieve a stable immune function, which has a significant effect on improving the inflammatory response [16].

MTX has an effect on T lymphocytes, reduces TCD8+ lymphocytes and other T cell functions, and inhibits neutral chemotaxis [17–20]. The effect of MTX on the treatment of psoriasis was retrospectively analyzed by Yu et al. [15]. Compared with MTX treatment, different doses of acitretin were more effective. The study results showed that the effective rates in the four groups were 69.1%, 86.9%, 88.2%, and 91.9%, respectively. The results of this study are highly consistent with those of Yu et al. This result shows that high-dose acitretin is more effective in the treatment of pustular psoriasis. Skin itching, dry skin, desquamation, chapped lips, elevated triglycerides, elevated cholesterol, and abnormal liver function, etc. are the main adverse reactions of acitretin, while the gastrointestinal discomfort, leukopenia, and abnormal liver function are the main adverse reactions of MTX. The study used MTX and acitretin for 52 weeks of continuous treatment and follow-up. The results of the study showed that the incidence of adverse reactions in the four groups were 16.2%, 8.1%, 10.3%, and 14.7%, respectively. When comparing with the MTX group, the different doses of acitretin group had relatively lower recurrence rates at 1 month and 3 months. The incidence of adverse reactions was higher in the high-dose group of acitretin, but it was fully tolerated by patients. The effective rate is relatively higher and the recurrence rate is relatively lower, so the treatment with a high dose of acitretin can be the optimal clinical plan. In addition, the study results showed that the improvement rates of GPPASI50 of the four groups were 71.4%, 78.3%, 80.2%, and 80.8%, respectively. The improvement rates of GPPASI75 in the four groups were 73.5%, 74.3%, 79.4%, and 80.9%, respectively. The improvement rates of GPPASI90 were 12.9%, 13.1%, 13.4%, and 13.8%, respectively. The results confirmed that the treatment with high-dose acitretin can reduce the severity of skin lesions in patients to a greater extent and can further shorten the time for erythema, fever, and pustules to resolve, thereby reducing the mental and psychological pressure of patients. Pustular psoriasis affects the health of patients to a large extent. After treatment with acitretin and MTX, the BSA and DLQI scores in the four groups were significantly reduced. And when comparing with the control group, the BSA and DLQI scores of the study group decreased more significantly (*P* < 0.05). The results confirmed that in terms of improving the life quality and reducing the severity of the disease, the treatment of high dose acitretin is of great significance, with high patient satisfaction and treatment compliance.

TLR7 activates NF-*κ*B through the MyD88-dependent pathway, triggers chemokines and inflammatory cytokines, and activates TGF-*β*-activated kinase 1 (TAK1), IL-1 receptor-associated kinase (IRAK), and TNF receptor-associated factor 6 (TRAF6). In patients with psoriasis, the expression of NF-*κ*B, TLR7, and MyD88 proteins in HK-2 cells increased after hypoxia and reoxygenation, which may aggravate the degree of cell damage. Under these conditions, the expression of NF-*κ*B and MyD88 protein was decreased and apoptosis was reduced after transfection with TLR7-SiRNA, which increased cell activity. Therefore, in this state, hypoxia and reoxygenation upregulated the TLR7 protein of HK-2 cells, activated the TLR7/MyD88/NF-*κ*B signaling pathway, and aggravated the damage of HK-2 cells. Overactivation of the TLR7/MyD88/NF-*κ*B signaling pathway is the main mechanism of aggravating HK-2 cell injury. Inhibition of TLR7 expression could block the TLR7/MyD88/NF-*κ*B signaling pathway, down-regulate the expression of NF-*κ*B and MyD88 proteins and alleviate cell damage. In conclusion, TLR7 plays an important role in HK-2 cells in the progression of disease, and the TLR7/MyD88/NF-*κ*B signaling pathway is involved in the hypoxia reoxygenation injury of HK-2 cells. Inhibition of TLR7 expression can alleviate the cytotoxic damage caused by hypoxia and reoxygenation, and the inflammatory response and oxidative stress indexes are significantly reduced, cell apoptosis is reduced, and the degree of hypoxia and reoxygenation damage is reduced, thus providing a new entry point for the clinical treatment of psoriasis. The results of this study also showed that the expression levels of TLR7 and CXCL16 were reduced after treatment with acitretin compared with MTX, especially in the high-dose acitretin group.

In summary, the clinical effect of the high dose of acitretin on pustular psoriasis is remarkable. It can reduce the recurrence rate and improve the quality of life and clinical symptoms. Therefore, a high dose of acitretin is worth popularizing and applying.

## Figures and Tables

**Figure 1:** Comparison of the improvement rates of GPPASI50, GPPASI75, and GPPASI90 with four groups.

**Figure 2:** Comparison of the BSA and DLQI scores with four groups.

**Figure 3:** Comparison of the incidence of adverse reactions with four groups.

**Figure 4:** Comparison of the treatment efficiency with four groups.

**Table 1:** Comparison of the time to symptom resolution in the four groups.

Group	Case quantity	Erythema resolution time (day)	Fever resolution time (day)	Pustules resolution time (day)
Control group	14	36.5 ± 4.3	4.5 ± 1.2	22.5 ± 3.4
Low-dose group	13	30.2 ± 3.8	4.1 ± 1.0	21.7 ± 3.2
Medium -dose group	13	28.6 ± 3.1	3.7 ± 0.8	20.3 ± 2.5
High-dose group	14	24.3 ± 2.7	3.2 ± 0.5	16.9 ± 2.1
*F*	/	17.524	14.635	15.781
*P*	/	<0.05	<0.05	<0.05

**Table 2:** Comparison of the recurrence rates of the four groups at 1 month and 3 months.

Group	Case quantity	Recurrence rate at 1 month		Recurrence rate at 3 months	
		Recurrence	Not recurrence	Recurrence	Not recurrence
Control group	14	3 (21.4)	11 (78.6)	3 (21.4)	11 (78.6)
Low-dose group	13	3 (23.1)	10 (76.9)	2 (15.4)	11 (84.6)
Medium-dose group	13	1 (7.7)	12 (92.3)	1 (7.7)	12 (92.3)
High-dose group	14	1 (7.1)	13 (92.9)	1 (7.1)	13 (92.9)
*F*	/	5.241		6.824	
*P*	/	<0.05		<0.05	

**Table 3:** The expression of CXCL16 and TLR7 in the four groups after treatment.

Group	Case quantity	CXCL16 (ng/L)	TLR7 (ng/L)
Control group	14	98.36 ± 12.64	56.31 ± 6.61
Low-dose group	13	84.32 ± 27.83	42.16 ± 20.53
Medium-dose group	13	77.14 ± 26.32	37.22 ± 18.16
High-dose group	14	48.25 ± 14.79	25.17 ± 12.37
*T*	/	9.16	10.21
*P*	/	<0.05	<0.05

## Data Availability

The data used to support the findings of this study are available from the corresponding author upon request.
